The article "Application of Intraoperative Electromyography Intelligent Monitoring in Orthopedic Surgery under General Anesthesia" was published in 2023. Journal: Contrast Media Mol Imaging.

# Application of Intraoperative Electromyography Intelligent Monitoring in Orthopedic Surgery under General Anesthesia

**DOI:** 10.1155/2023/1484802

**Published:** 2023-02-20

**Authors:** Mingmin Zhang, Junfeng Duan, Yanchun Chen, Chunyu Zhang

**Affiliations:** Department of Anesthesiology, Hangzhou Fuyang Hospital of Orthopedics of Traditional Chinese Medicine, Hangzhou, Zhejiang 311400, China

## Abstract

To study the application of intraoperative EMG intelligent monitoring in orthopedic surgery under general anesthesia, a total of 53 patients who underwent orthopedic surgery from February 2021 to February 2022 were selected. The combined monitoring of somatosensory evoked potential (SEP), motor evoked potential (MEP), and electromyography (EMG) was used to analyze the monitoring efficiency. In 38 of the 53 patients, the intraoperative signal was normal, and there was no postoperative neurological dysfunction; one case had abnormal signal, and the abnormality still existed after debugging, but no obvious neurological dysfunction was found after operation; the remaining 14 cases had abnormal signal. There were 13 early warnings in SEP monitoring; 12 early warnings in MEP monitoring; 10 early warnings in EMG monitoring. There were 15 cases of early warning in the joint monitoring of the three, and the sensitivity of the combined monitoring of SEP + MEP + EMG was significantly higher than that of the single monitoring of SEP, MEP, and EMG (*p* < 0.05). There was no significant difference in specificity, positive predictive value, and negative predictive value between combined monitoring and single monitoring (*p* > 0.05). The combined monitoring of EMG, MEP, and SEP in orthopedic surgery can significantly improve the safety of surgery, its sensitivity and negative predictive value were significantly higher than the monitoring effects of the two alone.

## 1. Introduction

The development of neurological deficits following spinal surgery is a complication with serious consequences, and some of these complications occur during surgery without any identifiable adverse event [1]. Back pain and symptoms of nerve root compression, including pain, numbness, and weakness, are common causes of disability and reduced overall quality of life. In most cases, initial conservative treatment, including rest, core muscle strengthening, and nonsteroidal anti-inflammatory drugs, helps with recovery [2]. However, surgical intervention is sometimes required to decompress nerve roots and restore spinal stability, posterior laminectomy, and discectomy can be used for isolated nerve root compression.

Although bone fusion is the preferred treatment for degenerative intervertebral disc disease, it will cause related nerve root compression, such as the nerve root associated with anterior displacement or spinal instability [3]. Recently, multimodal intraoperative neurophysiological monitoring (IONM), including somatosensory evoked potential (SEP), motor evoked potential (MEP), and electromyography EMG) has been used and has been shown to be effective in preventing nerve damage during spinal surgery. Somatosensory-evoked potential is a kind of neurophysiological examination, which can help doctors estimate the location, scope, degree, and prognosis of patients, and is widely used in various nervous system diseases. Motor-evoked potential (MEP) is a noninvasive detection method. MEP is a muscle motor complex potential recorded by stimulating the motor cortex in the contralateral target muscle; check the overall synchronization and integrity of motor nerve transmission and conduction pathways from the cortex to muscles. Electromyography is a technique that records the electrical activities of various electrophysiological characteristics of muscles in a quiet state, in a state of random contraction to varying degrees, and when peripheral nerves are stimulated after inserting concentric needle electrodes into muscles. EMG is a traditional neural monitoring technique that monitors resting electrical activity of muscles and is divided into real-time EMG and trigger electromyography (Trigger-EMG), SEP is used to monitor dorsal column function, and MEP monitors the function of the anterior and central spinal cord, including the corticospinal tract [4]. Since the introduction of ITOM, most studies have used signal loss as an alarm signal to indicate nerve damage, which may predict postoperative neurologic deterioration, but few studies have investigated the clinical significance of improvement in ITOM signaling during surgery. In this study, we analyzed the waveform changes of individual ITOM monitoring, such as SEP, MEP, and EMG, during orthopedic surgery, and compared the sensitivity and specificity of these monitoring methods to determine the best method which can be used to detect postoperative neurological deficits during surgery.

The article "Application of Intraoperative Electromyography Intelligent Monitoring in Orthopedic Surgery under General Anesthesia" was published in 2023. Journal: Contrast Media Mol Imaging.

## 2. Clinical Data

### 2.1. General Information

The total of 53 patients who underwent orthopedic surgery in our hospital from February 2021 to January 2022 were selected as the study subjects, including 34 males and 19 females; aged 45–78 years, with an average age of (59.04 ± 10.01 years); and the course of illness from 1 to 10 years, with an average (6.72 ± 2.20) years. All patients received joint SEP, MEP, and EMG monitoring during surgery and followed up for 3 months after surgery. The study was approved by the Ethics Committee of the Hospital and all patients had signed informed consent forms.

### 2.2. Inclusion Criteria [5]

The inclusion criteria include the following: ① patients with lumbar spinal stenosis, spinal spondylolisthesis, and degenerative lumbosacral spine disease requiring surgery; ② patients with instability, radiculopathy, or neurogenic claudication, which do not respond to conservative treatment or require unilateral neurodepression.

### 2.3. Exclusion Criteria

The exclusion criteria include the following: ① severe underlying or psychiatric disorders; ② cauda equina syndrome or active infection; ③ previous lumbar surgery, ozone intervention, or radiofrequency ablation; ④ bilateral nerve decompression; ⑤ bleeding disorders, coagulation abnormalities, or preoperative anemia; ⑥ unwillingness or inability to participate in treatment and completion of follow-up; ⑦ related electronic device implants; ⑧ unilateral or bilateral waveform deletions of SEP or MEP.

### 2.4. Surgical and Anesthetical Methods

Surgical methods include intervertebral fusion internal fixation, lumbar spinal stenosis initiation decompression graft fusion internal fixation, lumbar posterior incision and compound internal fixation, spinal canal enlargement decompression bone graft fusion internal fixation, and posterior pedicle nail internal fixation. Avoid the use of nondepolarizing neuromuscular blockers to reduce the potential confounding effects of exercise-induced responses. Use a limited (minimum alveolar concentration of volatile anesthetics less than 0.5) or whole-vein anesthetics that do not use volatile anesthetic gases to reduce any effect on somatosensory evoked potentials. Standard monitoring is performed in the operating room with intravenous fentanyl 200 *μ*g and lidocaine 100 mg. Induction of intravenous midazolam 0.04 mg/kg, propofol 2 mg/kg, sufentanil 0.5 *μ*g/kg, and cis-atracuridinium 0.2 mg/kg. Dizolcin 10 mg/kg intravenously, then maintained at an anesthetic dose of 1.0 ug/(kg·min), based on which dexmedetomidine was given intravenously at 0.5 *μ*g/kg for 10 minutes, followed by intravenous pumping of propofol 4 to 12 mg/(kg·h), sufentanil 0.6 *μ*g/(kg·h), and single additional cis-atracurium of cistroxurimium 0.1 mg/(kg·h).

### 2.5. Monitoring Methods

Continuous monitoring was carried out from the time the patient is placed on the operating table until the patient woke up from anesthesia, adjusting the stimulation amplitude according to the needs of each patient. MEP: transcranial MEP was recorded bilaterally from the medial femoral muscle, tibiatrium, and tresptomy muscle, the stimulation electrode was placed in the international 10–20 EEG system C3 and C4, and multiple sequences of 5 to 7 pulses were stimulated at a constant voltage (400–500 V) using the subcutaneous needle electrode, and the duration of each pulse was 200 to 400 ms. The stimulation interval for each stimulus sequence was 2.0 to 4.0 ms. Placed the recording electrode on the muscle innervated by the corresponding nerve root and recorded the complex muscle action potential caused by the stimulation. SEP: involved a stimulation electrode placed in the posterior tibial nerve (PTN) of the ankle joint, recording the cortical potential from a subcutaneous needle electrode attached to the standard skull position. The stimulation intensity ranged from 35 to 45 mA, the stimulation rate was 2 Hz, and an average of 160 to 300 tests were performed per trace. The response was recorded in a referenced manner from multiple electrodes with fixed, mainly recorded the P40 latency and amplitude of the double lower extremity SSEP. EMG: divided into trigger electromyography (trigger-EMG) and real-time electromyography (F-EMG). The former was discontinuous monitoring to determine the integrity of pedicle screws and identify adjacent neural structures, while the latter continuously monitors changed due to nerve root traction, compression, manipulation, and stimulation, as well as pedicle screw insertion injuries. Intraoperative EEG/MYO/Evoked Potential Measurement System is a product of Cadwell Company of Cadwell, USA, model: Cascade pro. The emulsion-evoked potential system is a product of Nestor Medical Instruments (Beijing) Co., Ltd., model: VikingQuest.

The article "Application of Intraoperative Electromyography Intelligent Monitoring in Orthopedic Surgery under General Anesthesia" was published in 2023. Journal: Contrast Media Mol Imaging.

### 2.6. Exception Handling

Early warning criteria [6–8]: intraoperative combined EMG, SEP, and MEP monitoring is used as a basis for treatment, and if the MEP amplitude decreases by more than 80%, the continuous explosive EMG phenomenon of EMG is compared, and the continuous recording is compared with the baseline trajectory, the SEP amplitude is reduced by at least 50% or the delay is increased by 10%. Any of the three monitoring abnormalities are regarded as early warning standards, immediately stop the operation, and dispose of as follows: ① test the evoked potential again to exclude false positive, if the repeated test is normal, the operation continues; if there is still an abnormal alarm, then dispose of it according to the follow-up plan. ② Exclude whether the electrode is improperly placed, or the wiring is off, and whether the parameters of the monitor are set appropriately. ③ After excluding the above factors, check the patient's anesthesia, whether there is a muscle relaxant or inhalation anesthesia, observe the patient's vital signs and blood oxygen saturation, and wash the surgical area with warm normal saline to observe whether the abnormal warning is lifted. If it has not been lifted, consider whether it is caused by improper surgical procedures. ④ Checking the surgical situation for nerve damage due to insertion of the inserts, and remove immediately if confirmed and give high-dose glucocorticoid shock treatment; if there is an abnormal warning in the process of decompression, it may indicate that nerve damage has occurred. If the warning persists for 20 minutes after intervention, consideration should be given to whether to terminate surgery as appropriate. Observing the occurrence of neurological dysfunction in patients after surgery, and comparing with preoperative whether there is aggravation or improvement, so as to distinguish the efficacy value of intraoperative monitoring.

The article "Application of Intraoperative Electromyography Intelligent Monitoring in Orthopedic Surgery under General Anesthesia" was published in 2023. Journal: Contrast Media Mol Imaging.

### 2.7. Observation Indicators

MEP: early warning standards for complete loss of waveform or 80% reduction in amplitude from baseline; SEP: comparison of continuous recording with baseline trajectory, reducing amplitude by at least 50% or increasing delay by 10% as alert criteria; EMG: continuous outbreak of muscle contraction, especially nerve-root-dominated muscles that may be surgically injured. Neurological examination before and after surgery, including an assessment of changes in limb muscle strength and sensation, neurological complications are defined as exacerbations of any new neurological symptoms or signs or preexisting signs that occur immediately after surgery and are of a transient or permanent nature. The final clinical evaluation will be carried out by a neurologist.

True positive (TP): changes in evoked potential (EP) are observed during wake-up testing or at the end of surgery, followed by the emergence of new neurological disorders; true negative (TN): during the entire procedure, the evoked potential changes within the normal range compared with the baseline value, and no neurological deterioration was seen after surgery; false negative (FN): the evoked potential is consistent with the baseline value throughout the procedure, but postoperative neurological examination reveals a new neurological defect; false positive (FP): a change in evoked potential (EP) that led to the adoption of appropriate measures and did not eliminate the alarm, but no new neurological defects were observed during the wake-up test and no new defects were found at the end of the procedure; other: when alarms exist, surgeons adjusting the surgical approach, alarms are eliminated, they are without new neurological defects after surgery, however, it is difficult to determine whether it is due to the alert after taking measures to avoid postoperative neurological defects. Sensitivity is defined as 100% × TP/(TP + FN), specificity is defined as TN/(TN + FP) × 100%, positive predictive value (PPV) is defined as TP/(TP + FP) × 100%, and negative predictive value (NPV) is defined as TN/(TN + FN) × 100%.

The article "Application of Intraoperative Electromyography Intelligent Monitoring in Orthopedic Surgery under General Anesthesia" was published in 2023. Journal: Contrast Media Mol Imaging.

### 2.8. Statistical Methods

The experimental data were analyzed by SPSS 26.0 statistical software; the measurement data was expressed in$\left(\bar{x}\pm s\right)$ the comparison took *t-*tested, and the counting data was expressed as an example or percentage, and used the *x*^*2*^ test; the difference between p < 0.05 was statistically significant.

## 3. Results

### 3.1. Intraoperative Signal Monitoring and Prognosis

Among the 53 patients, 38 patients had normal intraoperative signals and no neurological dysfunction after surgery, which was true negative; 1 case had signal abnormalities, and abnormalities still existed after debugging, but no obvious neurological dysfunction was seen after surgery, which was listed as false positives. The remaining 14 cases had signal abnormalities, among which the SEP amplitude decreased due to incorrect nail positioning is shown in Figure 1(a), and the SEP amplitude decreased due to the concussion of the spinal cord during surgery is shown in Figure 1(b). The decrease in MEP amplitude due to traction of the spinal cord during surgery is shown in Figure 2(a), and the partial disappearance of the MEP amplitude due to implantation is shown in Figure 2(b). There was no significant changes which were seen in the EMG image, see Figure 3.

### 3.2. Intraoperative Signal Abnormalities

Among the 53 patients, 13 cases of SEP monitoring were early warning, including 10 cases of true positive; 12 cases of MEP monitoring were early warning, of which 7 cases were true positive; 10 cases of EMG monitoring were early warning, and 7 cases were true positive; 15 cases of early warning were detected in the joint monitoring of the three, when 14 cases were true positive; for details, see Table 1.

### 3.3. Comparison of Specificity, Sensitivity, and Positive and Negative Predictive Values of Intraoperative Monitoring Methods

The sensitivity of SEP + MEP + EMG combined monitoring was significantly higher than that of SEP, MEP, and EMG single monitoring (*p* < 0.05), and there was no significant difference in specificity, positive predictive value, and negative predictive value (*p* > 0.05), see Table 2.

## 4. Discussion

The number of spinal surgeries each year is increasing rapidly, and surgeons are constantly looking for new ways to reduce costs and potential surgical complications, particularly iatrogenic spinal injuries [9]. Spinal cord iatrogenic injuries that occur during instrument manipulation are a major concern for the spine and spinal surgeons, and the need for intraoperative monitoring to assess spinal cord functional integrity becomes even more important as innovative devices are increasingly used in spinal surgery [10]. To monitor spinal cord integrity and potential iatrogenic injury, IONM of the spinal cord has become an important adjunct to neurosurgery and orthopedic spine surgery [1]. From the late 1970s onwards, early monitoring relied on evoked potentials such as SEP, but current multimodal IONM involves assessing changes in the MEP and EMG activity. These additional monitoring modalities provide feedback to the surgeon on possible spinal cord injury during surgery [11]. IONM is a useful tool for determining the extent of nerve damage and accurately locating lesions during peripheral nerve surgery, the representative IONM pattern used in peripheral nerve surgery is the neural action potential, which can assess the physiological continuity of the nerve, and the microkinesis test including induction of complex motor action potentials through direct nerve stimulation and muscle recording can also be used [12]. In peripheral nerve surgery, the application of IONM can immediately and reliably confirm the extent of nerve damage, similar to the results of Yu Chen [3] et al. studies, meaning that IONM can be used for purposes other than its primary use, i.e., monitoring adverse neurological events during surgery. Therefore, through case presentation recommendations, IONM can be used as a tool to predict postoperative prognosis and to support decision-making during surgery by providing neurophysiological information about neural connections.

The article "Application of Intraoperative Electromyography Intelligent Monitoring in Orthopedic Surgery under General Anesthesia" was published in 2023. Journal: Contrast Media Mol Imaging.

Although IONM is good for monitoring underlying nerve damage, the efficacy of IONM-induced potential changes has been inconsistent. For example, SEP has been shown to be effective in monitoring spinal cord function during cervical and thoracic spine surgery, but not for nerve root levels during lumbosacral surgery [13]. SEP can also be used to evaluate specific nerve roots, but it cannot detect immediate changes in iatrogenic injury. In terms of diagnostic value, SEP and MEP have shown high sensitivity and specificity in predicting neurological deficits after surgery for spinal deformities, but have no significant value in cervical disc surgery [14]. For transforaminal lumbar fusion surgery, only the benefits of monitoring EMG activity during pedicle screw insertion were explored, and EMG is not a test for neural integrity, so the detection of EMG in iatrogenic injuries is severely limited, but the use of other evoked potential changes to monitor potential postoperative neurological deficits in patients undergoing surgery is not well described [15, 16]. Orthopedic surgery stretches peripheral nerves, which can lead to temporary or permanent nerve damage [17]. This study illustrates the benefits of using ITOM during orthopedic surgery, SEP + MEP + EMG monitoring can improve monitoring efficiency, timely prediction of intraoperative adverse events, and thus reduce the impact of surgery on neurological function. Peripheral nerves may be directly damaged by machinery or heat, secondary to poor localization, ischemia or thrombosis, and due to traction stretching to increase intraarticular space. Since patients may also have hematomas or inflammatory neuropathy after surgery, in order to avoid possible postoperative neurological defects, nerve stretching time in patients sensitive to traction and ischemia will be minimized. This allows surgeons to confidently pull when no major SEP changes are detected, or to reduce the severity or duration of traction when an alarm is raised. Because somatosensory and motor evoked potentials have different sensitivities and specificities for identifying nerve damage, they provide maximum patient protection when used in combination.

The article "Application of Intraoperative Electromyography Intelligent Monitoring in Orthopedic Surgery under General Anesthesia" was published in 2023. Journal: Contrast Media Mol Imaging.

## 5. Conclusion

1. Of the 53 patients, 38 had normal intraoperative signals and no postoperative neurological dysfunction, all of which were negative; one case had abnormal signal and was still abnormal after debugging, but there was no obvious neurological dysfunction after operation, so it was classified as false positive. The remaining 14 cases had abnormal signals, in which SEP amplitude decreased due to wrong nail positioning and SEP amplitude decreased due to spinal cord concussion during operation. MEP amplitude caused by spinal cord traction decreased during operation, and MEP amplitude caused by implantation partially disappeared. There was no significant change in the EMG image. The combined use of the three can effectively avoid the shortcomings of a single method. The combination of the three can correctly identify the intraoperative EMG signals and quickly infer the possible causes of abnormalities. SEP, MEP, and EMG single monitoring have high sensitivity, specificity is low, cannot make accurate judgments, the patient's relevant nerve root compression performance pain symptoms cannot be fed back in time, the sensitivity of the combination of the three is 100%, specificity is 97.44%, research value is high, intraoperative EMG intelligent monitoring provides a more objective safety index for surgery, improves the safety of surgery, and effectively reduces the occurrence of nerve injury and complications in patients.
2. The sensitivity of sep + mep + emg combined monitoring was significantly higher than that of SEP, MEP, and EMG alone (*p* < 0.05), and there was no significant difference in specificity, positive predictive value, and negative predictive value (*p* > 0.05). Intraoperative EMG intelligent monitoring is more effective in orthopedic surgery under general anesthesia and can provide reference for clinical orthopedic surgery.

The article "Application of Intraoperative Electromyography Intelligent Monitoring in Orthopedic Surgery under General Anesthesia" was published in 2023. Journal: Contrast Media Mol Imaging.

## Figures and Tables

**Figure 1:** (a, b) The SEP wave amplitude drop map.

**Figure 2:** (a, b) MEP wave amplitude drop map.

**Figure 3:** MEP amplitude.

**Table 1:** Intraoperative signal abnormalities (*n*).

Monitoring methods		The number of examples	True positive	True negative	False positive	False negative
SEP	Normal	40	10	37	3	3
	Abnormal	13				

MEP	Normal	41	7	35	5	6
	Abnormal	12				

EMG	Normal	43	7	39	3	4
	Abnormal	10				

SEP + MEP + EMG	Normal	38	14	38	1	0
	Abnormal	15				

**Table 2:** Comparison of specificity, sensitivity, and positive and negative predictive values of intraoperative monitoring methods (%).

Monitoring methods	Sensitivity	Specificity	Positive predictive values	Negative predictive values
SEP	10/13 (76.92)	37/40 (92.50)	10/13 (76.92)	37/40 (92.50)
MEP	7/13 (53.85)	35/39 (89.74)	7/12 (58.33)	35/41 (85.37)
EMG	7/11 (63.64)	39/42 (92.86)	7/10 (70.00)	39/43 (90.70)
SEP + MEP + EMG	14/14 (100.00)	38/39 (97.44)	14/15 (93.33)	38/38 (100.00)
*x* ^*2*^	8.437	1.858	4.728	5.852
*p*	0.038	0.603	0.193	0.119

## Data Availability

The figures and tables used to support the findings of this study are included in the article.
